# Newcastle Disease Virus Fusion Protein Is the Major Contributor to Protective Immunity of Genotype-Matched Vaccine

This article has been retracted.

**DOI:** 10.1371/journal.pone.0074022

**Published:** 2013-08-28

**Authors:** Shin-Hee Kim, Nanchaya Wanasen, Anandan Paldurai, Sa Xiao, Peter L. Collins, Siba K. Samal

**Affiliations:** 1 Virginia-Maryland Regional College of Veterinary Medicine, University of Maryland, College Park, Maryland, United States of America; 2 Laboratory of Infectious Diseases, National Institute of Allergy and Infectious Diseases, Bethesda, Maryland, United States of America; Virginia Polytechnic Institute and State University, United States of America

## Abstract

Virulent strains of Newcastle disease virus (NDV) can cause devastating disease in chickens worldwide. Although the current vaccines are substantially effective, they do not completely prevent infection, virus shedding and disease. To produce genotype-matched vaccines, a full-genome reverse genetics system has been used to generate a recombinant virus in which the F protein cleavage site has been changed to that of avirulent vaccine virus. In the other strategy, the vaccines have been generated by replacing the F and HN genes of a commercial vaccine strain with those from a genotype-matched virus. However, the protective efficacy of a chimeric virus vaccine has not been directly compared with that of a full-genome virus vaccine developed by reverse genetics. Therefore, in this study, we evaluated the protective efficacy of genotype VII matched chimeric vaccines by generating three recombinant viruses based on avirulent LaSota (genotype II) strain in which the open reading frames (ORFs) encoding the F and HN proteins were replaced, individually or together, with those of the circulating and highly virulent Indonesian NDV strain Ban/010. The cleavage site of the Ban/010 F protein was mutated to the avirulent motif found in strain LaSota. *In vitro* growth characteristics and a pathogenicity test indicated that all three chimeric viruses retained the highly attenuated phenotype of the parental viruses. Immunization of chickens with chimeric and full-length genome VII vaccines followed by challenge with virulent Ban/010 or Texas GB (genotype II) virus demonstrated protection against clinical disease and death. However, only those chickens immunized with chimeric rLaSota expressing the F or F plus HN proteins of the Indonesian strain were efficiently protected against shedding of Ban/010 virus. Our findings showed that genotype-matched vaccines can provide protection to chickens by efficiently preventing spread of virus, primarily due to the F protein.

## Introduction

Newcastle disease (ND) is a highly contagious avian disease with worldwide distribution [1]. The causative agent, Newcastle disease virus (NDV), is a member of the genus *Avulavirus* in the family *Paramyxoviridae*. The genome of NDV consists of six transcriptional units (3′-N–P-M-F–HN-L-5′) [2]. The F and HN proteins form spike-like projections on the outer surface of the viral envelop and are the neutralizing and protective antigens of NDV. The F protein is synthesized as an inactive precursor (F0) that is cleaved by host cell protease into two biologically active F1 and F2 subunits [3]. The cleavage of the F protein is a prerequisite for virus entry and cell-to-cell fusion. The sequence of the F protein cleavage site is a well-characterized, major determinant of NDV pathogenicity in chickens. Homotypic interaction between the F and HN proteins is necessary for initiation of the fusion process [4,5].

All NDV strains belong to a single serotype [6,7]. However, genetic and antigenic diversity are recognized for NDV isolates, and the detection of progressive changes in strains isolated over successive years indicates that NDV is a continually evolving virus [8,9]. Based on genome length and sequence of the F gene, NDV strains have been classified into classes I (nine genotypes, 1-9) and II (eleven genotypes, I-XI). Class I strains are usually avirulent. A recent study also proposes that class I viruses comprise a single genotype, while class II contains 15 genetic groups including 10 previously established (I–IX, and XI) and five new genotypes (X, XII, XIII, XIV and XV) [10]. Class II contains both virulent and avirulent strains and the avirulent vaccine strains LaSota and B1 presently in worldwide use. Currently, the circulating strains associated with disease outbreaks worldwide predominantly are from genotypes V, VI, and VII of class II [11–14]. In contrast, the LaSota and B1 vaccine strains were isolated some 60 years ago and belong to genotype II in class II. Although the current vaccines offer substantial protection against disease, they do not completely prevent infection or virus shedding, and disease can occur in vaccinated birds [8,12]. Recent studies indicated that inactivated vaccines or live attenuated vaccines developed from currently circulating genotype strains had increased effectiveness against current virulent strains, particularly in preventing shedding of challenge virus [15,16].

Recently, we developed a reverse genetics system for a highly virulent NDV strain Banjarmasin/010/10 (Ban/010) that was isolated from diseased chickens during an outbreak in Indonesia in 2010 [17]. The Ban/010 virus is classified in genotype VII of class II and has only 89 and 87% amino acid identity for the F and HN proteins, respectively, with the LaSota and B1 vaccine strains [18]. A mutant virus, named recombinant Ban/AF (rBan/AF), was generated in which the virulent F protein cleavage site motif “RRQKR↓F” was modified to be identical to that of strain LaSota “GRQGR↓L” by three amino acid substitution (underlined) [17]. The rBan/AF virus was completely avirulent, and was genetically stable during 10 consecutive passages in chickens. Serological analysis showed that rBan/AF induced higher neutralization and hemagglutination inhibition antibody titers against the prevalent viruses than did the commercial vaccines B1 or LaSota. Both rBan/AF and the commercial vaccines provided protection against clinical disease and mortality after challenge with virulent NDV strain Ban/010 (genotype VII) or GB Texas (genotype II). However, rBan/AF significantly reduced challenge virus shedding from the vaccinated birds compared to the B1 vaccine.

These results confirm that a genotype-matched vaccine generated by reverse genetics can provide better protection than commercial vaccines [15–17]. However, development of a reverse genetics system for a circulating NDV strains can be costly and time consuming. An alternative strategy for producing genotype-matched vaccine is to replace the F and HN genes of a recombinant commercial vaccine strain with those of circulating strains in which the virulent F protein cleavage site motif was modified to an avirulent motif. Although this strategy is cost-effective and less time consuming, there are concerns that a chimeric virus may not be genetically stable and growth retarded due to gene incompatibility. Furthermore, a chimeric genotype-matched vaccine has never been directly compared with a same genotype-matched vaccine made by full-genome reverse genetics. Therefore, the purpose of this study was to compare the protective immunity of genotype VII vaccines developed by chimeric and by full-genome reverse genetics approaches. In order for this study, we generated three recombinant chimeric LaSota viruses in which the F and/or HN ORF was replaced with that of rBAN/AF, the attenuated version of Ban/010. These chimeric viruses were compared to the parental recombinant LaSota (rLaSota) and rBan/AF viruses for replication *in vivo* and *in vitro*, and for immunogenicity and protective efficacy against challenge with virulent GB Texas or Ban/010 viruses. This study also evaluated the relative contributions of F versus HN in the superior protection provided by vaccine virus that is homologous to the challenge virus. These results will be useful for development of genotype-matched NDV vaccines.

## Materials and Methods

### Viruses and cells

The chicken embryo fibroblast cell line (DF1) and human epidermoid carcinoma cell line (HEp-2; ATCC, Manassas, VA, USA) were grown in Dulbecco’s minimal essential medium (DMEM) with 10% fetal bovine serum (FBS) and maintained in DMEM with 5% FBS. The modified vaccinia virus strain Ankara (MVA) expressing T7 RNA polymerase was kindly provided by Dr. Bernard Moss (NIAID, NIH) and propagated in primary chicken embryo fibroblast cells in DMEM with 2% FBS. In experiments that required supplementations of exogenous protease for the cleavage of the F protein, normal SPF chicken egg allantoic fluid was added to a concentration of 10%.

NDV strains rLaSota [19] and rBan/AF [17] and the three recombinant chimeric viruses generated in this study were grown in the allantoic cavities of 9-day-old specific pathogen free (SPF) embryonated chicken eggs. Virus stocks were quantified by hemagglutination (HA) assay with chicken erythrocytes. All experiments involving virulent NDV were performed in our USDA approved enhanced Biosafety Level-3 (BSL-3+) facility following the guidelines and approval of the Animal Care and Use Committee (IACUC), University of Maryland. All experiments were approved by the IACUC (protocol number R-09-81) and conducted following the guidelines. All animal care and handling, including euthanasia were conducted according to the procedures of Animal Care and Use committee and guideline of the American Veterinary Medical Association. All efforts were made to minimize discomfort and pain. The personnel conducting this experiment examined infected birds three times a day for clinical symptoms following the well-established scoring system. Birds that show a total score of 0 were considered "normal" while birds showing scores of 1 to 8 were considered "sick." If a bird presents a score of 2 or 3 in any of the categories above, we increased the monitoring frequency to 3 times daily. Supportive care was provided for animals that show scores of 2 or 3. If the condition worsens or does not improve after it has reached a score of 3, it was euthanized as it is considered that the bird has reached a moribund state. If necessary, facility veterinarian in the department was contacted to determine whether the bird needs to be euthanized or requires supportive care. Supportive care was provided if it does not interfere with the objective of this study. Birds were anesthetized and killed by an overdose of isoflurane, the inhalant anesthetic. Briefly, sterile cotton gauze was placed in the bottom of a sterile bell jar and was covered with a wire mesh. Approximately, 1 to 2 ml of isoflurane was added into the cotton gauze. The bird was placed in the jar and the lid was closed quickly. The bird was removed from the jar after cessation of breathing.

### Generation of recombinant chimeric NDV strain LaSota in which the F and/or HN gene ORFs were replaced by those of the avirulent Indonesian strain rBan/AF

The F and HN ORFs of the avirulent strain rBan/AF were placed individually or together into a full-length antigenomic cDNA of NDV strain LaSota in place of the corresponding LaSota F and HN ORF(s) (Figure 1). These manipulations were facilitated by the presence of unique restriction enzyme sites (PacI, MluI, and AgeI) created in the untranslated regions (UTRs) flanking the F and HN ORFs in the NDV cDNA. The F and HN ORFs of rBan/AF were modified to be flanked by 5´ and 3´ UTRs of the respective rLaSota F or HN gene along with the compatible restriction enzyme sites by overlapping PCR. The engineered rBan/AF F and/or HN genes were digested with the appropriate restriction enzymes and used to replace the corresponding genes in the full-length LaSota cDNA, resulting in three full-length chimeric NDV cDNAs (Figure 1). Thus, the LaSota gene-start and gene-end signals flanking the F and HN genes remained undisturbed.

**Figure 1:** Construction and recovery of three chimeric versions of the LaSota vaccine strain in which the complete F and/or HN gene ORF was replaced with that of rBan/AF, an attenuated version of the circulating virulent Indonesian Ban/010 strain. (A) Genome maps of the parental rLaSota and rBan/AF strains and the three chimeric derivatives. ORFs are shown as rectangles that are filled for those derived from rLaSota and are open for those from rBan/AF. The F protein cleavage sites are shown. (B) SDS-PAGE analysis of purified virions of strains rLaSota (lane 1), Ban/AF (lane 2), rLaSota-Ban/AF F (lane 3), rLaSota-Ban/AF HN (lane 4), and rLaSota-Ban/AF F HN (lane 5). The viruses were harvested from allantoic fluids, purified through a 30% sucrose cushion, and analyzed on an 8% SDS-PAGE gel under reducing conditions, and stained with Coomassie brilliant blue.

Infectious viruses were generated using a reverse genetics system established in our laboratory [20]. Briefly, HEp-2 cells were transfected with three plasmids individually encoding the N, P, and L proteins (2.0 µg, 1.0 µg, and 0.5 µg per single well of a six-well dish, respectively) and a fourth plasmid encoding the full-length antigenome (5.0 µg) using Lipofectamine (Invitrogen) and simultaneously infected with vaccinia MVA expressing T7 RNA polymerase at a multiplicity of infection (MOI) of 1 PFU/cell. Two days after transfection, alloquot of transfection mixture was inoculated into the allantoic cavity of 9-day-old embryonated chicken eggs. Following incubation for 2 days, allantoic fluid was harvested and recovery of the virus was confirmed by hemagglutination assay using 1% chicken red blood cells. The recovered viruses were plaque purified. The absence of adventitious mutations in the F and/or HN genes of Indonesian strain in the recovered viruses were confirmed by nucleotide sequencing analysis using primers targeting a downstream of the M gene and an upstream of the L gene.

### Cleavage of the F protein of chimeric viruses

To evaluate cleavage of the F proteins of the chimeric viruses, DF1 cells were infected at an MOI of 0.1, and cell lysates were collected at 24 h post-infection (hpi), denatured under reducing conditions, subjected to electrophoresis on an 8% polyacrylamide gel, and subjected to Western blot analysis separately with anti-NDV F rabbit polyclonal antiserum [21] and an anti-NDV HN monoclonal antibody.

### Growth characteristics of parental and chimeric NDVs in DF1 cells

The ability of the chimeric viruses to produce plaques was tested in DF1 cells under 0.8% methylcellulose overlay. The plaques were immunostained using polyclonal antibody raised against the N protein of NDV [22]. The multicycle growth kinetics of the F and HN chimeric viruses, along with their respective parental viruses, was evaluated in DF1 cells in the presence of 10% chicken egg allantoic fluid. Virus titers in the collected supernatants were quantified in DF1 cells by limiting dilution in the presence of added allantoic fluid and expressed as 50% tissue culture infectious dose (TCID_50_/ml) by the end-point method of Reed and Muench [23].

### Mean death time in embryonated chicken eggs

The pathogenicity of parental and chimeric viruses was determined by the mean death time (MDT) test in 9-day-old SPF embryonated chicken eggs [1]. Briefly, a series of 10-fold dilutions of infected allantoic fluid (0.1 ml) was inoculated into the allantoic cavities of five 9-day-old eggs per dilution and incubated at 37 °C. The eggs were examined once every 8 h for 7 days, and the time of embryo death was recorded. The MDT was determined as mean time (h) for the minimum lethal dose of virus to kill all the inoculated embryos. The criteria for classifying the virulence of NDV isolates are: <60 h, virulent strains; 60 to 90 h, intermediate virulent strains; and >90 h, avirulent strains.

### Immunization of chickens with parental and chimeric NDVs

Two-week-old SPF chickens in groups of eleven (11 birds each) were immunized with each virus (200 µl of each, 10^6^ EID_50_) by the intranasal route. One group of chickens remained as unvaccinated controls. Three birds from each group were sacrificed at 4 days post-infection (dpi) and tissues samples (lung and trachea) were collected for vaccine virus titration. Virus titers were determined by limiting dilution and immunostaining in DF1 cells as described before. The presence of virus in the tissue samples also were determined by inoculation into 9-day-old SPF embryonated chicken eggs, which provides a more sensitive means of detection but does not provide a titer. In general, we obtained HA titers ranging from 2^4^ to 2^7^ from positive samples. At 3 dpi, the allantoic fluids were tested for virus growth by HA assay. For analysis of antibody responses, serum samples (3 ml from each chicken) were collected on weeks 2, 3, 4, and 5. Serum antibody titers were determined by hemagglutination inhibition (HI) assay using rLaSota or rBan/AF as antigen [17].

### Challenge of immunized chickens with virulent NDV strains

Five weeks post immunization, the remaining chickens (eight per immunizing virus) were transferred to a USDA-certified BSL3containment facility for NDV challenge. The birds in each group were challenged with 100 chicken 50% lethal dose (CLD_50_) of virulent NDV strains GB-Texas (four birds) or Ban/010 (four birds) through the oculo-nasal route [17]. Oral and cloacal swabs were collected from three birds at 4 and 7 dpi, and shedding of the challenge virus was determined by inoculating clarified swab samples into 9-day-old SPF embryonated chicken eggs and conducting HA assay as described above. Three chickens from each group were sacrificed at 4 days post-challenge (dpc) to evaluate challenge virus replication in different organs. Tissue samples (brain, trachea, lungs, and spleen) were collected, and the challenge virus titers in homogenized tissue samples were determined by a limiting end point dilution assay as described above.

### Statistical Analysis

Statistically significant differences in serological analysis between different immunized chicken groups were evaluated by one-way analysis of variance (ANOVA) (SPSS 13.0 for Windows, SPSS Inc, Chicago, IL).

## Results

### Generation of recombinant chimeric LaSota viruses with the F and/or HN gene ORF replaced by that of a circulating Indonesian NDV strain

We used reverse genetics to make three chimeric derivatives of the LaSota vaccine strain in which the complete ORF of the F and/or HN genes was replaced with that of the rBan/AF strain (Figure 1A), which is a version of the highly virulent Ban/010 strain that was rendered avirulent solely by three amino acid substitutions in the cleavage site of the F protein. Specifically, the F protein cleavage site of rBan/AF, and of the three chimeric viruses, was identical to that of strain LaSota. Infectious viruses were recovered from all of the three chimeric cDNAs (rLaSota-Ban F, rLaSota-Ban HN, and rLaSota-Ban F HN). To evaluate genetic stability, the viruses were passaged five times in 9-day-old embryonated chicken eggs. All the viruses were able to replicate well in the eggs (> 2^8^ HAU/ml) and the sequences of the F and HN genes were confirmed, showing that the introduced ORFs were maintained without any adventitious mutations.

We further evaluated incorporation of heterologous glycoproteins into chimeric virions, since the presence of the compatible cytoplasmic tails and transmembrane regions is important for NDV replication [24]. The viral proteins in partially purified parental and chimeric viruses [25] were analyzed by SDS-PAGE and visualized by Coomassie blue staining (Figure 1B). This confirmed a similar pattern of the major structural proteins into each virus, with the expected sizes and amounts, suggesting that the substitutions in rLaSota backbone did not affect virion assembly (Figure 1B).

### Syncytium formation and cleavage efficiency of the F protein of chimeric viruses in vitro

Strain LaSota lacks a polybasic sequence or furin motif at the F protein cleavage site, and depends on extracellular protease for cleavage [19]. In our previous study, we modified the highly virulent Indonesian Ban/010 strain by changing its cleavage site sequence (R RQK R↓F) to that of LaSota (GRQGR↓L), resulting in the avirulent rBan/AF derivative. Whereas the Ban/010 parent induced extensive syncytia and plaque formation in cell culture in the absence of added protease, the rBan/AF derivative caused only single-cell infections without syncytia or plaques in the presence or absence of extracellular protease [17]. Therefore, in the present study, the ability of the chimeric viruses to form syncytia and plaques in cell culture was determined. DF1 cells were infected with the parental (rLaSota and rBan/AF) and the three chimeric viruses at an MOI of 0.01 in the presence or absence of 10% allantoic fluid as protease supplementation. The cells were visualized 48 hpi by photomicroscopy directly (Figure 2A) and following immunostaining with antiserum against the NDV N protein (Figure 2B). In parallel, the ability of the viruses to produce plaques was evaluated on DF1 cells under 0.8% methylcellulose overlay (not shown). In the presence of added protease, the rLaSota virus produced syncytia (Figure 2A and B) and plaques (not shown), whereas the rBan/AF virus produced neither. Among the three chimeric viruses, only the one containing F from the LaSota and HN from the rBan/AF strain (rLaSota-Ban/AF HN) produced syncytia and plaques, similar to those of rLaSota. In contrast, the other two chimeric viruses (rLaSota-Ban/AF F and rLaSota-Ban/AF F HN) produced neither syncytia (Figure 2A and B) nor plaques (not shown). Thus, the formation of syncytia and plaques in the presence of protease was associated with the presence of the LaSota F protein. Evaluation of the cleavage efficiency of the F proteins by Western blot analysis showed that the LaSota-derived F protein present in both rLaSota and rLaSota-Ban/AF HN was cleaved more efficiently than the rBan/AF-derived F protein present in the other viruses (Figure 3). These results suggest that the greater efficiency of cleavage of the LaSota-derived F protein was required for syncytium and plaque formation.

**Figure 2:** Production of syncytia by parental and chimeric viruses. DF1 cells in six-well plates were infected with the indicated viruses at a multiplicity of infection (MOI) of 0.01 PFU/cell, incubated for 72 h, and visualized by photomicroscopy directly (A) or following immunoperoxidase staining using antiserum against the N protein of NDV, with viral antigen stained red (B).

**Figure 3:** Cleavage of the F0 proteins of parental and chimeric viruses. (A) Proteolytic cleavage of the F0 proteins of parental and chimeric viruses in infected DF1 cells analyzed by Western blot. (B) The positions of the precursor protein F0, the cleavage product F1, and the HN protein are indicated. Lanes: 1. rLaSota, 2. rBan/AF, 3. rLaSota-Ban/AF F, 4. rLaSota-Ban/AF HN, and 5. rLaSota-Ban/AF F HN (B) The relative levels of the F0 and F1 proteins in the Western blot experiment in part C were measured by Bio-Rad Gel Image analysis, and the efficiency of cleavage was determined by dividing the amount of F1 by the amount of F1 plus F0. Each bar represents mean and standard error of the mean of triplicate samples.

### Growth characterization of chimeric NDVs in vitro

The growth kinetics of parental and chimeric NDVs was evaluated in DF1 cells after infection at an MO1 of 0.01 in the presence of exogenous protease (Figure 4). Parental rLaSota replicated more efficiently than rBan/AF in the first 24 h of infection, but the titers were similar thereafter. Among the chimeric viruses, rLaSota-Ban/AF HN grew to higher titer than the two parental viruses and the other two chimeric viruses, reaching a maximum titer of 1.3 × 10^7^ TCID_50_/ml at 40 hpi. The other two chimeric viruses (rLaSota-Ban/AF F and rLaSota-Ban/AF F HN) replicated less efficiently than the other tested viruses and reached their maximum titers (10^6^ TCID_50_/ml) at 56 hpi. The pattern of *in vitro* replication of chimeric viruses also showed the correlation with their ability to form syncytia in DF1 cells (Figure 2).

**Figure 4:** *In vitro* multicycle growth of parental and chimeric viruses in chicken embryo fibroblast DF1 cells following infection with an MOI of 0.01 PFU/cell. Exogenous protease was provided in the infected cells. The viral titers were determined by limiting dilution on DF1 cells.

### Pathogenicity of the chimeric viruses

The pathogenicity of chimeric viruses was evaluated by a standard, internationally-accepted pathogenicity test for NDV, namely the MDT assay in embryonated chicken eggs (Table 1). Of the two parental viruses, rBan/AF (122 h) was somewhat more attenuated than the rLaSota virus (112 h). For the three chimeric viruses, the order of increasing attenuation was rLaSota-Ban/AF HN (129 h), rLaSota-Ban/AF F (148 h), and rBan/AF F HN (>168 h). Thus, introduction of either of the two rBan/AF glycoproteins conferred attenuation, with F having a greater effect than HN, and the effect was greatest when both rBan/AF glycoproteins were introduced. At least in the case of the rBan/AF HN glycoprotein, this attenuation was not due to a direct defect in the replication of the chimeric virus, since the chimeric rLaSota-Ban/AF HN virus replicated the most efficiently in cell culture (Figure 4).

**Table 1:** Pathogenicity of parental and chimeric viruses in embryonated eggs.

Virus	MDT (h)^a^
rLaSota	112
rBan/AF	122
rLaSota-Ban/AF F	148
RLaSota-Ban/AF HN	129
rLaSota-Ban/AF F HN	>168

^a^ Mean embryo death time (MDT): the mean time (h) for the minimum lethal dose of virus to kill all of the inoculated embryos. Pathotype definition: virulent strains, <60 h; intermediate virulent strains, 60 to 90 h; avirulent strains, >90 h.

### Replication, immunogenicity, and protective efficacy of chimeric NDVs

To evaluate the protective efficacy of the chimeric viruses, 2-week-old chickens were immunized with each virus by intranasal route. Three birds from each group were sacrificed at 4 dpi and tissue samples (brain, trachea, lungs, and spleen) were collected for virus titration. Virus titration of the homogenates by limiting dilution assay showed that detection of parental and chimeric viruses was restricted to the trachea, and their titers were low, ranging from 1.6 to 2.4 log_10_ TCID_50_/g, with slight differences between the parental and chimeric viruses (data not shown). To enhance the sensitivity of virus detection, the tissue homogenates also were inoculated into eggs (Table 2). Replication of rLaSota and rBan/AF was confirmed in the trachea and lungs, whereas replication of the three chimeric viruses was mostly found in the trachea of the immunized birds. None of the viruses were detected in the brain and spleen.

**Table 2:** Replication of parental and chimeric viruses in 2-week-old immunized chickens.

	Virus replication in embryonated eggs^a^			
Virus	Brain	Trachea	Lung	Spleen
rLaSota	0/3	3/3	2/3	0/3
rBan/AF	0/3	3/3	2/3	0/3
rLaSota-Ban/AF F	0/3	3/3	0/3	0/3
rLaSota-Ban/AF HN	0/3	3/3	1/3	0/3
rLaSota-Ban/AF F HN	0/3	3/3	1/3	0/3

^a^ Groups of 2-week-old chickens were inoculated with each virus by the intranasal route. Three birds from each group were sacrificed on day 4, and tissues samples (brain, trachea, lung, and spleen) were collected and homogenized. To confirm the virus replication, each sample (100 µl, containing approximately 10 µg of tissue) of homogenized tissue was inoculated into each of three eggs, and allantoic fluids were collected on 3 dpi. Virus replication was determined by hemagglutination assay.

The immunogenicity of the chimeric viruses was determined by collecting sera at 2, 3, 4, and 5 weeks post-immunization and evaluating antibody responses using HI assay (log_2_) against the two different parental viruses, namely the rLaSota (Figure 5A) and rBan/AF (Figure 5B) strains. The highest titers were obtained from sera collected at 2 (rBan/AF-specific assay) or 4 (rLaSota-specific assay) weeks post-immunization, after which the titers decreased. In the rLaSota-specific assay, antisera raised against either parental virus tended to have higher HI titers than those raised against the chimeric viruses, especially at 2 weeks post-immunization. In the rBan/AF-specific assay, antisera raised against the parental rBan/AF virus generally had the highest titers at the various time points, whereas antisera against the parental rLaSota virus generally had the lowest titers. Among the sera raised against the three chimeric viruses, there was no clear pattern of reactivity associated with the presence of the homologous versus the heterologous HN protein.

**Figure 5:** Induction of serum antibodies in 2-week-old chickens in response to infection with parental and chimeric viruses. Chickens were inoculated with each virus (64 HA units) by the intranasal route in the same experiment as Table 2. Sera were collected at 2, 3, 4, and 5 weeks post-infection. Virus-specific antibodies were measured by a hemagglutination inhibition assay using rLaSota (A) or rBan/AF (B) virus and chicken erythrocytes.

To evaluate the protective efficacy of chimeric NDVs, at 5 weeks post-immunization, the remaining immunized chickens in each immunization group were divided into two challenge groups. Each challenge group (8 birds each) was challenged with 100 CLD_50_ per chicken of the virulent GB Texas (genotype II, homologous to the LaSota vaccine) or the virulent wild-type Indonesian strain (Ban/010, genotype VII, the parent of the rBan/AF strain) via the oculo-nasal route. In addition, three chickens each from the unimmunized group were challenged with either of the two challenge NDVs. For the unimmunized chickens, challenge with the GB Texas virus resulted in clinical symptoms (at 4 day post-challenge (dpc), and 100% of mortality at 5 dpc, whereas challenge with the Ban/010 virus resulted in 100% of mortality at 3 dpc (data not shown). The virus titers in the trachea of dead chickens were >7.0 log_10_ TCID_50_/g. In contrast, all of the previously-immunized chickens (5 chickens for each group) were completely protected from clinical disease and mortality against the GB-Texas and Ban/010 strains.

Shedding and replication of the GB-Texas and Ban/010 challenge viruses in the immunized chickens were evaluated. Oral and cloacal swabs (3 birds each) were collected at 4 and 7 dpc and inoculated into eggs for sensitive detection of infectious virus. In addition, 3 birds from each challenge group were sacrificed at 4 dpi and tissue samples (brain, trachea, lungs, and spleen) were collected and tissue homogenates prepared. These were evaluated for the presence of virus by inoculation into eggs, and virus titers were determined by limiting dilution assay, as above. In the GB-Texas challenged groups, virus shedding was not detected in most swab samples (Table 3), and no virus was detected in any of the collected tissue samples (data not shown). This indicated that all the immunized groups of the chickens were efficiently protected against GB-Texas. However, in the Ban/010-challenged group, virus shedding was detected in both the oral and cloacal swabs in all of the chickens immunized with rLaSota (Table 3), and high virus titers were detected in the trachea (2.9 × 10^6^ TCID_50_/g) and lungs (1.8 × 10^5^ TCID_50_/g) (Figure 6). Similarly, virus shedding was detected in chickens immunized with rLaSota containing the Ban/AF HN (rLaSota-Ban/AF HN). In contrast, virus shedding was present in only 1 of 3 in chickens immunized with a genotype-matched vaccine, rBan/AF, and only in the oral swab. At 7 dpi, no oral or coacal shedding of challenge viruses was detected in all of the collected swab samples (data not shown).

**Table 3:** Oral and cloacal shedding of NDV challenge viruses.

	NDV strain GBT challenge		NDV strain Indonesia challenge	
Chicken group^a^	Oral	Cloacal	Oral	Cloacal
rLaSota	0/3	0/3	3/3	3/3
rBan/AF	1/3	0/3	1/3	0/3
rLaSota-Ban/AF F	1/3	0/3	0/3	0/3
rLaSota-Ban/AF HN	1/3	0/3	3/3	2/3
rLaSota-Ban/AF F HN	0/3	0/3	1/3	0/3

^a^ Groups of 2-week-old chickens were inoculated with each virus by the intranasal routes and challenged with NDV strain GBT or Indonesia. Oral (A) and cloacal (B) swabs were collected from the 3 birds in each group on day 4 and 7 post challenge. To confirm the shedding of challenge virus, aliquots (100 µl each, out of a total of 1 ml of swab fluid) of the collected samples were inoculated into three eggs, and allantoic fluids were collected on 3 dpi. Virus replication was determined by hemagglutination assay. On day 7 post challenge, challenge virus shedding was not detected in all of the collected samples.

**Figure 6:** Shedding of challenge Ban/010 virus in chickens previously immunized with parental and chimeric viruses. From the challenge experiment in Table 3, tissue samples were harvested from the 3 birds in each group on day 4 post-challenge, and virus titers were determined by a limiting dilution assay on DF-1 cells. Data from challenge with the GB Texas strain are not shown because no virus was detected.

The two chimeric LaSota viruses containing rBan/AF F and F and HN together showed comparable levels of protective efficacy to that of rBan/AF. Our findings showed that rBan/AF vaccine and the two chimeric viruses containing the genotype-matched F gene (rLaSota-Ban/AF F and rLaSota-Ban/AF F HN) effectively prevented shedding of Indonesian challenge virus, whereas viruses lacking the Indonesian F gene, namely rLaSota and chimeric rLaSota-Ban/AF HN, were less effective in preventing shedding of Indonesian challenge virus. These results show that the genotype-matched vaccines provide better protection than genotype mismatched vaccines, and this superior efficacy is due to the F protein.

## Discussion

All NDV isolates belong to a single serotype. Consistent with this, currently used vaccines, such as strains B1 and LaSota, are known to protect against morbidity and mortality caused by NDV isolates in different parts of the world [26]. However, recent studies have suggested that NDV strains currently in circulation represent genotypes that differ from that of the vaccine strains [8], and the current vaccines allow considerable breakthrough infection, shedding, and disease by the presently circulating genotype viruses. Infection and shedding permits recirculation of the virus in the environment and provides a setting in which the viral population may acquire mutations and adaptive changes in response to immune pressure [27]. Therefore, the use of genotype-matched vaccines has been suggested for better control of NDV [15,16,28]. Our previous study also demonstrated that an attenuated vaccine virus (rBan/AF) generated by reverse genetics from a circulating virulent virus in Indonesia provided better protection against genotype-matched isolates than that provided by the genotype-mismatched vaccine stains LaSota and B1 [17]. However, generation of a genotype-matched vaccine by reverse genetics can be time consuming. Therefore, in this study, we generated recombinant chimeric viruses, using an existing LaSota-based reverse genetics system, by replacing the ORF of F and HN genes of LaSota with those from rBan/AF, which is a recombinant attenuated derivative of the highly virulent Indonesian Ban/010 strain of genotype VII. The attenuated phenotype of the rBan/AF strain was derived solely by the introduction of three amino acid substitutions in the F protein cleavage site of the virulent Ban/010 parent, which changed the site to be identical to that of the LaSota strain.

In our study, all the chimeric viruses were readily recovered, and the incorporation of the surface glycoproteins into virions and the yield of virions were similar between parental and chimeric viruses. This indicated that the amino acid sequence differences between the F and HN proteins of rLaSota versus rBan/AF did not detectably affect virus assembly and recovery. However, in *vitro* characterization of the parental and chimeric viruses showed that the F protein of the LaSota strain was cleaved more efficiently, in the presence of added allantoic fluid as a source of protease, than the F protein of rBan/AF, and the presence of this protein was associated with the formation of syncytia and plaques as well as better growth *in vitro*. This was true for both the parental and chimeric viruses. Thus, the rBan/AF HN virus had efficient cleavage of the F protein, induced syncytium and plaque formation, and had relatively efficient replication in DF1 cells, similar to rLaSota. Nonetheless, the virus was somewhat more attenuated (MDT 129 h) than rLaSota (MDT 112 h). In contrast, rLaSota-Ban/AF F and rLaSota-Ban/AF F HN showed inefficient cleavage of the F protein, single cell infection without syncytium or plaque formation, and reduced replication in infected DF1 cells. The finding that cleavage of the rBan/AF F protein was less efficient than that of the rLaSota F protein, even though their cleavage activation sequences were identical, indicated that structural features of the rBan/AF F protein additional to the cleavage site affect proteolytic processing of the F protein. Chimeric LaSota containing rBan/AF F and HN together resulted in a greater attenuation of the virus *in ovo* (MDT > 168 h) than either glycoprotein alone, showing that the rBan/AF HN protein also contributed to attenuation *in ovo*. One possible explanation could be that the glycoproteins from rBan/AF may not be perfectly compatible with the LaSota background. However, this did not appear to be true for the rBan/AF HN protein, at least, since the rLaSota-Ban/AF HN virus replicated more efficiently *in vitro* than either parent, and thus did not appear to be impaired.

Immunization of 2-week-old chickens confirmed that all the chimeric viruses were highly attenuated. Replication of the three chimeric viruses was mostly limited to the trachea (Table 2), and thus they were somewhat more attenuated in birds than the LaSota vaccine strain, consistent with the results of the MDT assay. Thus, they should be safe vaccines. Despite this attenuation, the chimeric viruses induced relatively good serum antibody responses. In general, sera from chickens immunized with parental and chimeric viruses had higher HI titers against rLaSota than rBan/AF (p<0.05). This was associated with greater restriction of the GB-Texas challenge strain (homologous to LaSota) compared to the Ban/010 challenge strain. In the Ban/AF-specific HI assay, the highest HI titers were observed with parental rBan/AF, followed by rLaSota containing rBan/AF F protein (rLaSota-Ban/AF F), whereas the lowest titers were observed with rLaSota (p<0.05). Our challenge study showed that chickens vaccinated by rLaSota-Ban/AF F and rLaSota-Ban/AF F HN completely prevented shedding of the Ban/010 challenge virus, whereas rLaSota-Ban/AF HN did not prevent shedding of Ban/010 (Figure 5B). Thus, the presence of the rBan/AF F protein in the immunizing virus was associated with complete restriction of the Ban/010 challenge virus. It is noteworthy that this greater efficacy was not associated with more efficient replication *in vitro* (in fact, the rLaSota-Ban/AF F and rLaSota-Ban/AF F HN viruses replicated less efficiently *in vitro* than the others; Figure 4) or *in vivo* (Table 2). These results indicate that, although the F and HN proteins of NDV are known to be the virus neutralizing antigens and the major protective antigens [29–31], the presence of the homologous F protein was more important in restricting the homologous challenge virus.

Previously, cross protection studies have suggested that chickens vaccinated with a live LaSota vaccine displayed disease symptoms after being challenged with antigenic variants of genotype VII [32]. Inactivated vaccines and live attenuated vaccines developed from currently circulating genotype strains were shown to have increased effectiveness in preventing virus shedding [15,16]. In contrast, several studies showed that current vaccines have good protective efficacy for morbidity and mortality against viruses circulating in Asia [33,34]. However, shedding of challenge virus was not evaluated in these studies. It has been thought that the extent of the vaccine failure in the commercial farm group may be due to poor vaccination practices, field environmental and/or immunosuppressive factors affecting the efficacy of the vaccine [35]. However, our previous study with the Ban/010 strain circulating in Indonesia suggested that complete prevention of shedding of genotype VII can be achieved by a recombinant genotype matched vaccine generated by reverse genetics [17]. In the present study, evaluation of recombinant chimeric viruses confirmed our previous findings that a genotype-matched vaccine generated either by chimeric or full-genome approach is needed for prevention of virus shedding. Further our study identified the F protein as the major protective antigen for efficient protection of chickens against genotype VII NDV strain. This study also needs to be verified by evaluating protective efficacy in broiler chickens, which are older (slaughtered at 5-16 weeks).

## References

[1] AlexanderDJ (1989) Newcastle disease, In: PurchaseHGArpLHDomermuthCHPearsonJE A laboratory manual for the isolation and identification of avian pathogens, 3rd ed. The American Association of Avian Pathologists, Kendall/Hunt Publishing Company pp. 114-120.

[2] LambR, ParksG (2007) Paramyxoviridae: the viruses and their replication, In: KnipeDMHowleyPMGriffinDELambRAMartinMA Philadelphia: Lippincott Williams & Wilkins pp. 1449–1496.

[3] LambRA, PatersonRG, JardetzkyTS (2006) Paramyxovirus membrane fusion: lessons from the F and HN atomic structures. Virology 344: 30-37. doi:10.1016/j.virol.2005.09.007. PubMed: 16364733.1636473310.1016/j.virol.2005.09.007PMC7172328

[4] DengRZ, WangA, MirzaM, IorioRM (1995) Localization of a domain on the paramyxovirus attachment protein required for the promotion of cellular fusion by its homologous fusion protein spike. Virology 209: 457-469. doi:10.1006/viro.1995.1278. PubMed: 7778280.777828010.1006/viro.1995.1278

[5] MelansonVR, IorioRM (2004) Amino acid substitutions in the F-specific domain in the stalk of the Newcastle disease virus HN protein modulate fusion and interfere with its interaction with the F protein. J Virol 78: 13053-13061. doi:10.1128/JVI.78.23.13053-13061.2004. PubMed: 15542657.1554265710.1128/JVI.78.23.13053-13061.2004PMC525001

[6] PedersenJC, SenneDA, WoolcockPR, KindeH, KingDJ et al. (2004) Phylogenetic relationships among virulent Newcastle disease virus isolates from the 2002-2003 outbreak in California and other recent outbreaks in North America. J Clin Microbiol 42: 2329-2334. doi:10.1128/JCM.42.5.2329-2334.2004. PubMed: 15131226.1513122610.1128/JCM.42.5.2329-2334.2004PMC404648

[7] SamalSK (2011) Newcastle disease and related avian paramyxoviruses, In: SamalSK The biology of paramyxoviruses. Caister Academic Press pp. 69-114.

[8] MillerPJ, DecaniniEL, AfonsoCL (2010) Newcastle disease: evolution of genotypes and the related diagnostic challenges. Infect Genet Evol 10: 26-35. doi:10.1016/j.meegid.2009.09.012. PubMed: 19800028.1980002810.1016/j.meegid.2009.09.012

[9] KimSH, NayakS, PalduraiA, NayakB, SamuelA et al. (2012) Complete genome sequence of a novel Newcastle disease virus strain isolated from a chicken in West Africa. J Virol 86: 11394-11395. doi:10.1128/JVI.01922-12. PubMed: 22997417.2299741710.1128/JVI.01922-12PMC3457136

[10] DielDG, da SilvaLHA, LiuH, WangZ, MillerPJ et al. (2012) Genetic diversity of avian paramyxovirus type 1: Proposal for a unified nomenclature and classification system of Newcastle disease virus genotypes. Infect Genet Evol 12: 1770-1779. doi:10.1016/j.meegid.2012.07.012. PubMed: 22892200.2289220010.1016/j.meegid.2012.07.012

[11] AldousEW, FullerCM, MynnJK, AlexanderDJ (2004) A molecular epidemiological investigation of isolates of the variant avian paramyxovirus type 1 virus (PPMV-1) responsible for the 1978 to present panzootic in pigeons. Avian Pathol 33: 258-269. doi:10.1080/0307945042000195768. PubMed: 15276997.1527699710.1080/0307945042000195768

[12] CattoliG et al. (2010) Emergence of a new genetic lineage of Newcastle disease virus in West and Cwntral Africa-implications for diagnosis and control. Vet Micobiol 142: 168-176.10.1016/j.vetmic.2009.09.06319939590

[13] KhanST, Rehmani, RueC, MillerP, AfonsoCL (2010) Phylogenetic and pathological characterization of Newcastle disease virus isolates from Pakistan. J Clin Microbiol 48: 1892–1894. doi:10.1128/JCM.00148-10. PubMed: 20237105.2023710510.1128/JCM.00148-10PMC2863937

[14] LiuXF, WanHQ, NiXX, WuYT, LiuWB (2003) Pathotypical and genotypical characterization of strains of Newcastle disease virus isolated from outbreaks in chicken and goose flocks in some regions of China during 1985–2001. Arch Virol 148: 1387–1403. PubMed: 12827467.1282746710.1007/s00705-003-0014-z

[15] MillerPJ, KingDJ, AfonsoCL, SuarezDL (2007) Antigenic differences among Newcastle disease virus strains of different genotypes used in vaccine formulation affect viral shedding after a virulent challenge. Vaccine 25: 7238–7246. doi:10.1016/j.vaccine.2007.07.017. PubMed: 17719150.1771915010.1016/j.vaccine.2007.07.017

[16] MillerPJ, EstevezC, YuQ, SuarezDL, KingDK (2009) Comparison of viral shedding following vaccination with inactivated and live Newcastle disease vaccines formulated with wild-type and recombinant viruses. Avian Dis 53: 39–49. doi:10.1637/8407-071208-Reg.1. PubMed: 19432002.1943200210.1637/8407-071208-Reg.1

[17] XiaoS, NayakB, SamuelA, PalduraiA, Kanabagattebasavarajappa M, et al. (2012) Generation by reverse genetics of an effective, stable, live-attenuated Newcastle disease virus vaccine based on a currently circulating, highly virulent Indonesian strain. PLOS ONE 7: e52751

[18] XiaoS, PalduraiA, NayakB, SamuelA, BharotoEE et al. (2012) Complete genome sequences of Newcastle disease virus strains circulating in chicken populations of Indonesia. J Virol 86: 5969-5970. doi:10.1128/JVI.00546-12. PubMed: 22532534.2253253410.1128/JVI.00546-12PMC3347286

[19] HuangZ, KrishnamurthyS, PandaA, SamalSK (2001) High-level expression of a foreign gene from the 3´ proximal first locus of a recombinant Newcastle disease virus. J Gen Virol 82: 1729-1736. PubMed: 11413385.1141338510.1099/0022-1317-82-7-1729

[20] KrishnamurthyS, HuangZ, SamalSK (2000) Recovery of a virulent strain of Newcastle disease virus from cloned cDNA: expression of a foreign gene results in growth retardation and attenuation. Virology 278: 168-182. doi:10.1006/viro.2000.0618. PubMed: 11112492.1111249210.1006/viro.2000.0618

[21] SamalS, KumarS, KhattarSK, SamalSK (2011) A single amino acid change Q114R in cleavage site sequence of Newcastle disease virus fusion protein attenuates viral replication and pathogennicity. J Gen Virol 92: 2333-2338. doi:10.1099/vir.0.033399-0. PubMed: 21677091.2167709110.1099/vir.0.033399-0

[22] KimSH, XiaoS, ShiveH, CollinsPL, SamalSK (2012) Replication, neurotropism, and pathogenicity of avian paramyxovirus serotypes 1-9 in chickens and ducks. PLOS ONE 7: e34927. doi:10.1371/journal.pone.0034927. PubMed: 22558104.2255810410.1371/journal.pone.0034927PMC3340391

[23] ReedLJ, MuenchHA (1938) A simple method of estimating fifty percent endpoints. Am J Hyg 27: 493-497.

[24] KimSH, SubbiahM, SamuelAS, CollinsPL, SamalSK (2011) Roles of the fusion and hemagglutinin-neuraminidase proteins in replication, tropism, and pathogenicity of avian paramyxoviruses. J Virol 85: 8582-8596. doi:10.1128/JVI.00652-11. PubMed: 21680512.2168051210.1128/JVI.00652-11PMC3165810

[25] PeterHD, RobinsonWS (1965) Isolation of the Newcastle disease virus. Proc Natl Acad Sci U S A 54: 794-800. doi:10.1073/pnas.54.3.794. PubMed: 5217460.521746010.1073/pnas.54.3.794PMC219746

[26] ChoSH, KwonHJ, KimTE, KimJH, YooHS et al. (2008) Characterization of a recombinant Newcastle disease vaccine strain. Clin Vaccine Immunol 15: 1572–1579. doi:10.1128/CVI.00156-08. PubMed: 18768673.1876867310.1128/CVI.00156-08PMC2565930

[27] PerozoF, MarcanoR, AfonsoCL (2012) Biological and Phylogenetic Characterization of a Genotype VII Newcastle Disease Virus from Venezuela: Efficacy of Field Vaccination. J Clin Microbiol 50: 1204-1208. doi:10.1128/JCM.06506-11. PubMed: 22238433.2223843310.1128/JCM.06506-11PMC3318500

[28] HuS, MaH, WuY, LiuW, WangX et al. (2009) vaccine candidate of attenuated genotype VII Newcastle disease virus generated by reverse genetics. Vaccine 27: 904-910. doi:10.1016/j.vaccine.2008.11.091. PubMed: 19095026.1909502610.1016/j.vaccine.2008.11.091

[29] BoursnellME et al. (1990) A recombinant fowlpox virus expressing the hemagglutinin-neuraminidase gene of Newcastle disease virus (NDV) protects chickens against challenge by NDV. Virology 78: 297–300. PubMed: 2167557.10.1016/0042-6822(90)90408-j2167557

[30] CossetFL et al. (1991) Newcastle disease virus (NDV) vaccine based on immunization with avian cells expressing the NDV hemagglutinin-neuraminidase glycoprotein. Virology 185: 862–866. doi:10.1016/0042-6822(91)90560-X. PubMed: 1660204.166020410.1016/0042-6822(91)90560-x

[31] KaracaK et al. (1998) Recombinant fowlpox viruses coexpressing chicken type I IFN and Newcastle disease virus HN and F genes: influence of IFN on protective efficacy and humoral responses of chickens following in ovo or post-hatch administration of recombinant viruses. Vaccine 16: 1496–1503. doi:10.1016/S0264-410X(97)00295-8. PubMed: 9711795.971179510.1016/s0264-410x(97)00295-8

[32] QinZM, TanLT, XuHY, MaBC, WangYL et al. (2008) Pathotypical characterization and molecular epidemiology of Newcastle disease virus isolates from different hosts in China from 1996 to 2005 J. Clin Microbiol 46: 601-611. doi:10.1128/JCM.01356-07.10.1128/JCM.01356-07PMC223812118077643

[33] JeonWJ, LeeEK, LeeYJ, JeongOM, KimYJ et al. (2008) Protective efficacy of commercial inactivated Newcastle disease virus vaccines in chickens against a recent Korean epizootic strain. J Vet Sci 9: 295-300. doi:10.4142/jvs.2008.9.3.295. PubMed: 18716450.1871645010.4142/jvs.2008.9.3.295PMC2811842

[34] LiuXF, WanHQ, NiXX, WuYT, LiuWB (2003) Pathotypical and genotypical characterization of strains of Newcastle disease virus isolated from outbreaks in chicken and goose flocks in some regions of China during 1985–2001. Arch Virol 148: 1387–1403. PubMed: 12827467.1282746710.1007/s00705-003-0014-z

[35] DortmansJC, PeetersBP, KochG (2012) Newcastle disease virus outbreaks: vaccine mismatch or inadequate a p p l i c a t i o n ? Vet Microbiol 160: 17-22. doi:10.1016/j.vetmic.2012.05.003. PubMed: 22655976.2265597610.1016/j.vetmic.2012.05.003

[36] MossB, Elroy-SteinO, MizukamiT, AlexanderWA, FuerstTR (1990) Product review. New mammalian expression vectors. Nature 348: 91–92. doi:10.1038/348091a0. PubMed: 2234068.223406810.1038/348091a0

